The article "An immunoinformatics and extended molecular dynamics approach for designing a polyvalent vaccine against multiple strains of Human T-lymphotropic virus (HTLV)" was retracted in 2025. Reasons: unreliable results or conclusions; concerns about the peer review; concerns about the article.

# An immunoinformatics and extended molecular dynamics approach for designing a polyvalent vaccine against multiple strains of Human T-lymphotropic virus (HTLV)

**DOI:** 10.1371/journal.pone.0287416

**Published:** 2023-09-08

**Authors:** Abu Tayab Moin, Nurul Amin Rani, Md. Asad Ullah, Rajesh B. Patil, Tanjin Barketullah Robin, Nafisa Nawal, Talha Zubair, Syed Iftakhar Mahamud, Mohammad Najmul Sakib, Nafisa Nawal Islam, Md. Abdul Khaleque, Nurul Absar, Abdullah Mohammad Shohael

**Affiliations:** 1 Faculty of Biological Sciences, Department of Genetic Engineering and Biotechnology, University of Chittagong, Chattogram, Bangladesh; 2 Faculty of Biotechnology and Genetic Engineering, Sylhet Agricultural University, Sylhet, Bangladesh; 3 Faculty of Biological Sciences, Department of Biotechnology and Genetic Engineering, Jahangirnagar University, Savar, Dhaka, Bangladesh; 4 Department of Pharmaceutical Chemistry, Sinhgad Technical Education Society’s, Sinhgad College of Pharmacy, Maharashtra, India; 5 Notre Dame College, Dhaka, Bangladesh; 6 Faculty of Biological Sciences, Department of Microbiology, University of Chittagong, Chattogram, Bangladesh; 7 Department of Biochemistry and Microbiology, North South University, Bashundhara, Dhaka, Bangladesh; 8 Faculty of Basic Medical and Pharmaceutical Sciences, Department of Biochemistry and Biotechnology, University of Science & Technology Chittagong, Khulshi, Chittagong, Bangladesh; The Islamia University of Bahawalpur Pakistan, PAKISTAN

## Abstract

Human T-lymphotropic virus (HTLV), a group of retroviruses belonging to the oncovirus family, has long been associated with various inflammatory and immunosuppressive disorders. At present, there is no approved vaccine capable of effectively combating all the highly pathogenic strains of HTLV that makes this group of viruses a potential threat to human health. To combat the devastating impact of any potential future outbreak caused by this virus group, our study employed a reverse vaccinology approach to design a novel polyvalent vaccine targeting the highly virulent subtypes of HTLV. Moreover, we comprehensively analyzed the molecular interactions between the designed vaccine and corresponding Toll-like receptors (TLRs), providing valuable insights for future research on preventing and managing HTLV-related diseases and any possible outbreaks. The vaccine was designed by focusing on the envelope glycoprotein gp62, a crucial protein involved in the infectious process and immune mechanisms of HTLV inside the human body. Epitope mapping identified T cell and B cell epitopes with low binding energies, ensuring their immunogenicity and safety. Linkers and adjuvants were incorporated to enhance the vaccine’s stability, antigenicity, and immunogenicity. Initially, two vaccine constructs were formulated, and among them, vaccine construct-2 exhibited superior solubility and structural stability. Molecular docking analyses also revealed strong binding affinity between the vaccine construct-2 and both targeted TLR2 and TLR4. Molecular dynamics simulations demonstrated enhanced stability, compactness, and consistent hydrogen bonding within TLR-vaccine complexes, suggesting a strong binding affinity. The stability of the complexes was further corroborated by contact, free energy, structure, and MM-PBSA analyses. Consequently, our research proposes a vaccine targeting multiple HTLV subtypes, offering valuable insights into the molecular interactions between the vaccine and TLRs. These findings should contribute to developing effective preventive and treatment approaches against HTLV-related diseases and preventing possible outbreaks. However, future research should focus on in-depth validation through experimental studies to confirm the interactions identified *in silico* and to evaluate the vaccine’s efficacy in relevant animal models and, eventually, in clinical trials.

The article "An immunoinformatics and extended molecular dynamics approach for designing a polyvalent vaccine against multiple strains of Human T-lymphotropic virus (HTLV)" was retracted in 2025. Reasons: unreliable results or conclusions; concerns about the peer review; concerns about the article.

## 1. Introduction

Human T-lymphotropic viruses (HTLV) belong to the human retroviruses family, specifically in the genus Deltaretrovirus, and they infect the human body, leading to various diseases such as adult T-cell leukemia (ATL). HTLV-1, HTLV-2, HTLV-3, and HTLV-4 are the four major subtypes of HTLV identified to date. These group of viruses not only cause malignancy but also other inflammatory and immunosuppressive diseases [1,2]. HTLVs are enveloped viruses with a diameter ranging from 80 to 100 nm and within the HTLV virions, the reverse transcriptase (RT), integrase, protease viral enzymes, and capsid proteins form complexes with the two covalently bonded genomic RNA strands [3,4]. The proviral genome of HTLVs is approximately 9kb in length and is flanked by 5’ and 3’ long terminal repeats (LTRs), which consist of U3, R, and U5 regions. These regions facilitate viral integration into the host genome and contain promoter elements with regulatory sequences for viral transcription [5,6].

Among the four major subtypes of HTLV identified to date, the pathogenic roles of HTLV-1 and HTLV-2 in the human body are well-studied to date compared to HTLV-3 and HTLV-4. This group of viruses are transmitted through bodily fluids like semen, blood and milk [2]. HTLV-1, in particular, is the most life-threatening member of this viral family, causing fatal ATL in approximately 5% of the infected cases that characterizes high blood circulation, lymph node swelling and immunosuppression [7,8]. Of the 4 types of ATL, acute ATL is most aggressive form of leukemia that results in median survival of patients less than one year. Moreover, this specific strain can also cause HTLV-1-associated myelopathy/tropical spastic paraparesis (HAM/TSP) that results in the progressive weakness of both legs and 50% of untreated patients are expected to lose their ability to walk within 10 years of initial diagnosis. HTLV-2 was first detected in a patient with hairy cell leukaemia and is considered less pathogenic when compared to HTLV-1 [9]. HTLV-2 has arguably been associated with developing HAM/TSP in infected patients like HTLV1 [10]. Moreover, HTLV-2 was also found to be associated with the onset of neuropathic disorders, including meningitis and chronic inflammatory demyelinating polyneuropathy (CIDP) and affecting patients clinical outcome negatively [11,12]. The global impact of HTLV-1 and HTLV-2 infections is alarming, with an estimated 5–10 million people infected worldwide [13]. HTLV-1 is highly prevalent in indigenous populations in Japan and South America, while HTLV-2 is primarily found in Central and South America [14].

The article "An immunoinformatics and extended molecular dynamics approach for designing a polyvalent vaccine against multiple strains of Human T-lymphotropic virus (HTLV)" was retracted in 2025. Reasons: unreliable results or conclusions; concerns about the peer review; concerns about the article.

HTLV-3 and HTLV-4 have been reported in isolated forest areas in the Republic of Cameroon. Despite exhibiting a similar genomic composition and ancestral relationship with HTLV-1 and HTLV-2, their potential risk to human health is still under investigation [15,16]. Furthermore, studies have revealed that subtle genomic reconstruction of HTLV-3 can lead to the production of virulent particles in the virus strain [17], indicating that the potential pathogenic roles of HTLV-3 and HTLV-4 should not be entirely overlooked.

Despite the HTLV-related diseases possess higher threat to the global public health, these group of diseases remain highly underrepresented in terms of developing an effective countermeasure through robust scientific research. HTLV-associated malignancies are often treated with conventional chemotherapy, bone marrow transplantation or monoclonal antibodies but these approaches often result in poor outcome [8]. Additionally, although there is some antiretroviral therapy which has shown some efficacy in suppressing viral replication of HTLVs, currently, there is no licensed vaccine available for HTLVs that may aid in curing a mass-infected population during any possible outbreaks or epidemics [18].

However, developing a vaccine against HTLVs has been challenging due to the ability of the virus to integrate its genetic material into the host genome, making it difficult to target with a vaccine. Additionally, the presence of a few distinct viral proteins that interfere with the immune system and the variability of the virus further complicate vaccine development [11,19]. Hence, developing a vaccine targeting the effective virulent protein against HTLVs is crucial due to their intricate mechanism of infection and evading the host defense system. Studies suggest that candidates able to boost anti-HTLV-envelope-glycoprotein antibodies may have potential roles in combating HTLV infection [20].

The article "An immunoinformatics and extended molecular dynamics approach for designing a polyvalent vaccine against multiple strains of Human T-lymphotropic virus (HTLV)" was retracted in 2025. Reasons: unreliable results or conclusions; concerns about the peer review; concerns about the article.

In this study, the Envelope Glycoprotein GP62 of the viruses was targeted as a potential antigen for designing the subunit vaccine. Glycoproteins, located on the outer layer of the viral envelope, are easily recognized by the immune system. The enveloped glycoprotein, which is a surface protein (SU) of HTLV attaches the virus to the host cell by binding to its receptor, while the transmembrane protein (TM) undergoes a conformational change upon interacting with the host cell, activating its fusogenic potential and leading to membrane fusion at the host cell plasma membrane. This fusion process allows the viral nucleocapsid to enter the cytoplasm of the host cell [21,22].

Finally, the aim of the study is to design an effective polyvalent subunit vaccine against the major causative agents of HTLV-related diseases i.e., HTLV-1, HTLV-2 using high-throughput bioinformatics strategies. Additionally, given that the pathogenic mechanism and virulence of other subtypes i.e., HTLV-3 remain under investigation, we also incorporated HTLV-3 subtype in our experimental design. However, since the virulent protein sequence of HTLV-4 is not yet reported in public repository, we didn’t consider HTLV-4 in our study. Despite the challenges in vaccine development, this research aims to provide molecular insights into how the designed subunit vaccine may counteract viral infections. The results obtained from this study will facilitate further in vitro and in vivo validation, advancing the understanding and potential implementation of the HTLV vaccines.

## 2. Methods

The stepwise methodology of the entire study is depicted in **S1 Fig in S1 File** as a flowchart.

### 2.1. Strain and protein selection with biophysical property analyses

From NCBI (https://www.ncbi.nlm.nih.gov/) database, three distinct HTLV strains, namely, HTLV-1, HTLV-2, and HTLV-3, were identified, and a virulent protein named Envelope glycoprotein gp62 was chosen for further epitope mapping. The target protein sequences of the chosen strains were then retrieved in FASTA format from the UniProt database (https://www.uniprot.org). The chosen protein sequence was then uploaded to the online antigenicity tool VaxiJen v2.0 (http://vaxijen/VaxiJen/VaxiJen.html) to examine the antigenic property [23]. Transmembrane topology was evaluated by using the TMHMM-2.0 server (https://services.healthtech.dtu.dk/service.php?TMHMM-2.0). By using the ExPASy ProtParam server (https://web.expasy.org/protparam//), we examined various physicochemical characteristics of the protein [24]. To find the conservancy pattern, the homologous sequence sets of the selected antigenic proteins were obtained from the NCBI database using the BLASTp program.

The article "An immunoinformatics and extended molecular dynamics approach for designing a polyvalent vaccine against multiple strains of Human T-lymphotropic virus (HTLV)" was retracted in 2025. Reasons: unreliable results or conclusions; concerns about the peer review; concerns about the article.

### 2.2. Epitope mapping analyses and vaccine construction

We utilized the Immune Epitope Database (IEDB) online tool (https://www.iedb.org/) to predict T-cell and B-cell epitopes of selected protein sequences, while keeping the default parameters. The full reference set of human leukocyte antigen (HLA) alleles was selected to predict MHC class I-restricted CD8+ cytotoxic T-lymphocyte (CTL) epitopes using the NetMHCpan EL 4.0 prediction method suggested by IEDB (http://tools.iedb.org/mhci/) [25]. For MHC class II-restricted CD4+ helper T-lymphocyte (HTL) epitopes, we used the IEDB-recommended 2.22 prediction method with the full reference set of HLA alleles (http://tools.iedb.org/mhcii/). To predict linear B-cell epitopes (LBL) of the chosen protein, we used the BepiPred technique 2.0 with the default parameters (http://tools.iedb.org/bcell/), and selected the highest-scoring LBL epitopes as prospective candidates for further analysis.

After the initial epitope prediction, we determined epitope antigenicity using the VaxiJen v2.0 server, predicted transmembrane topology using the TMHMM 2.0 server, and assessed allergenicity using the AllergenFP (https://ddg-pharmfac.net/AllergenFP/) and AllerTOP (https://www.ddg-pharmfac.net/AllerTOP/) servers. We also evaluated toxicity using the ToxinPred server (http://crdd.osdd.net/raghava/toxinpred/) [26]. The HTL epitopes’ capacity to induce IFN-g, IL-4, and IL-10 was predicted using the IFNepitope (http://crdd.osdd.net/raghava/ifnepitope/), IL4pred (http://crdd.osdd.net/raghava/il4pred/), and IL10pred (http://crdd.osdd.net/raghava/IL-10pred/) servers, respectively [27–29]. In addition, the epitopes’ conservancy was evaluated by generating a multiple sequence alignment using version 3.0 of the CLC Drug Discovery Workbench 3 software [30]. Epitopes with the highest potential for vaccine construction, based on their high antigenicity, non-toxicity, non-allergenicity, and conservancy, were chosen. To create the vaccine, these epitopes were combined with adjuvants like PADRE and human beta-defensin (hBds), and selective linkers such as EAAAK, AAY, and GPGPG.

### 2.3. Analyses of the biophysical and structural properties of the vaccine

To ensure the safety and efficacy of the vaccine, antigenicity and allergenicity analyses were conducted. The solubility of the vaccine construct upon expression in *Escherichia coli* was evaluated using the Protein-Sol server (https://protein-sol.manchester.ac.uk/) [31]. The biophysical characteristics of the vaccine constructions, including isoelectric pH, aliphatic and instability index, GRAVY values, hydropathicity, anticipated half-life, and other characteristics were assessed using the ProtParam tool of the ExPASy server. The secondary structure of the final multi-epitope vaccine was predicted using two servers, SOPMA (https://npsa-prabi.ibcp.fr/cgi-bin/npsa_automat.pl?page=/NPSA/npsa_sopma.html) and PSIPRED (http://bioinf.cs.ucl.ac.uk/psipred/) [32]. The trRosetta server (https://yanglab.nankai.edu.cn/trRosetta/) was used to modulate the tertiary structure of the vaccine constructs [33,34], which was later refined by the GalaxyRefine module of the GalaxyWEB server (http://galaxy.seoklab.org/) [35]. The improved models were then validated through the PROCHECK server (https://saves.mbi.ucla.edu/) for Ramachandran plots and ERRAT score plots. The Z score plots were generated using the ProSA-web server (https://prosa.services.came.sbg.ac.at/prosa.php) [36–38].

The article "An immunoinformatics and extended molecular dynamics approach for designing a polyvalent vaccine against multiple strains of Human T-lymphotropic virus (HTLV)" was retracted in 2025. Reasons: unreliable results or conclusions; concerns about the peer review; concerns about the article.

### 2.4. Molecular docking analyses

Initially, a molecular docking analysis was conducted to investigate the binding affinity between the CTL epitopes and HLA alleles. For the docking study with T cell epitopes, HLA-A*11:01 and HLA-DRB1*04:01 were selected. The PEP-FOLD Peptide Structure Prediction server was used to generate the 3D structures of the best CTL epitopes. The H-dock server (http://hdock.phys.hust.edu.cn/) was then utilized to perform the molecular docking analysis, demonstrating that the proposed epitopes could interact with at least one MHC molecule with minimum binding energy [39–41]. Subsequently, another molecular docking analysis was carried out between the vaccine constructs and TLR2 and TLR4 receptors to predict their binding affinities and interaction patterns. The TLR2 and TLR4 receptor structures were obtained from the RCSB PDB database, and the refined 3D structure of the multi-epitope construct served as the ligand. The binding affinity between the vaccine construct and TLR2 and TLR4 was calculated using the ClusPro 2.0 server and H-dock server (https://cluspro.bu.edu/login.php) [42]. The best-docked complex was identified based on the lowest energy-weighted score and docking efficiency.

### 2.5. Molecular dynamics simulation studies

The docked complexes of respective vaccine constructs with TLR2 and TLR4 were subjected to 100 ns molecular dynamics (MD) simulations with Gromacs 2020.4 [43] package using the resources of HPC cluster at Bioinformatics Resources and Applications Facility (BRAF), C-DAC, Pune. TLR2 and TLR4 have four chains each and the topologies for these chains and vaccine chains were prepared using the CHARMM-36 force field parameters [44,45]. The complexes of TLR2 and TLR4 with respective vaccine constructs were solvated with the TIP3P water model [46] after positioning them in a box of dodecahedron unit cells, keeping the boundary of system 1 nm from the edges of the box. The charges on each solvated system were neutralized where the TLR2 complex and the TLR4 complex required the addition of 8 and 16 sodium counter-ions, respectively. Further, the energy minimization was performed with the steepest descent algorithm employing the force constant threshold of 100 kJ mol^-1^ nm^-1^. The equilibration of each system for 1 ns was then carried out at constant volume and constant temperature (NVT) conditions where the temperature of 300 K was achieved with a modified Berendsen thermostat [47] and at constant volume and constant pressure (NPT) conditions where 1 atm pressure was achieved with Berendsen barostat [48]. The production phase MD simulations of 100 ns were performed on each equilibrated system without any restraints on the chain of TLR2 and TLR4. During production phase, MD simulations the temperature was held constant with a modified Berendensen thermostat, and pressure was held constant with a Parrinello-Rahman barostat [49]. However, the covalent bonds were restrained with the LINCS algorithm [50]. The long-range electrostatic energies were computed with Particle Mesh Ewald (PME) method [51]) with the cut-off of 1.2 nm. The trajectories from the production run were treated for removing the periodic boundary conditions (PBC) and then used in the analysis. The root mean square deviations (RMSD) from initial equilibrated positions of C-α atoms of each chain of TLRs and respective vaccine chains was investigated to gauge the stability of respective complexes. The fluctuations in the side chain atoms of each residue of TLR chains and vaccine chain was analyzed as root mean square fluctuation (RMSF) in each chain of systems. The compactness of system and consequent stability of system was analyzed in terms of radius of gyration (Rg) for each chain of TLRs and vaccine chain. The hydrogen bonds formed between vaccine chain and the TLR chains were analyzed using appropriate index files of respective chains. Further, the hydrogen bonds formed between vaccine and TLR chains were visually inspected using ChimeraX interface in equilibrated trajectory and trajectory extracted at 25, 50, 75 and 100 ns simulation time. Using the gmx_mdmat program the smallest distance between residues pairs for both the complexes were analyzed and used to obtain the residue wise contact maps [52]. Principal component analysis (PCA) [53] was performed to study the major path of motions where the program gmx_covar was employed to obtain a covariance matrix for the C-α atom of each complexes. This covariance matrix was diagonalized using gmx_anaeig program to get the eigenvectors and eigenvalues, where eigenvectors shows the path of motion while the eigenvalues show the mean square fluctuation. The first two principal components (PC1 and PC2) were in Gibb’s free energy landscape (Gibb’s FEL) analysis [54] using gmx sham program. In Gibb’s FEL the deep valleys represent the lowest energy states while the boundaries between the deep valleys show intermediate conformations of the systems. The secondary structural changes were analyzed from definition of protein secondary structure (DSSP) program [55,56]. Further, the extent to which the fluctuations and displacements of a side chains of each TLR chains and vaccine chain are correlated with one another was analyzed from dynamical cross-correlation matrix (DCCM) [56]. Poisson Boltzmann surface area continuum solvation (MM-PBSA) calculation [57,58] were performed to derive the binding free energy estimates between TLR chain and vaccine chain. However, as there are four larger chains in each TLRs and as MM-PBSA calculations are quite extensive, only 10 trajectories which were extracted at each 10 ns from MD simulation run were employed. The protein structures were rendered in ChimeraX [59], PyMOL [60], and VMD [57] and graphs were plotted in XMGRACE [58] interface, while the Gibb’s FEL plots were generated using python based Matplotlib package [61]. The DCCM analysis was performed in R statistical program [62] using Bio3D package [63].

The article "An immunoinformatics and extended molecular dynamics approach for designing a polyvalent vaccine against multiple strains of Human T-lymphotropic virus (HTLV)" was retracted in 2025. Reasons: unreliable results or conclusions; concerns about the peer review; concerns about the article.

### 2.6. Disulfide engineering and *in silico* cloning studies

Vaccine protein disulfide engineering was performed using the Disulfide by Design 2 server (http://cptweb.cpt.wayne.edu/DbD2/) to investigate the conformational stability of folded proteins. Throughout the analysis, the Cα-Cβ-Sγ angle was kept at its default value of 114.6° ± 10, and the χ3 angle was set at -87° or +97°. Residue pairs with energies lower than 2.5 Kcal/mol were chosen and converted to cysteine residues to form disulfide bridges [64]. During the in silico cloning study of the vaccine construct, the E. coli strain K12 was selected as the host. However, since the codon usage in humans and E. coli differs, the codon adaptation tool JCAT (http://www.jcat.de) was utilized to adapt the codon usage of the vaccine construct to well-characterized prokaryotic organisms in order to enhance the expression rate [65]. When using the JCAT server, it is important to avoid prokaryotic ribosome binding sites, BglII and Apa1 cleavage sites, and Rho independent transcription termination sites. The optimum sequence of the vaccine construct was then inverted, followed by conjugation of the N- and C-terminal BglII and Apa1 restriction sites using the SnapGene Software [66].

## 3. Results

### 3.1. Strain and protein selection with biophysical property analyses

The protein sequences of the target protein (Envelope glycoprotein gp62) in FASTA format were retrieved from the UniProt database. **Table 1** lists the UniProt accession numbers of the selected protein sequences. All the selected proteins were highly antigenic, stable, and have desirable physicochemical properties as listed in **S1 Table in S1 File.**

**Table 1:** List of the proteins used in this study with their UniProt accession numbers.

Strain	Isolate No.	Name of the protein	UniProt accession no.
HTLV-1	01	Envelope glycoprotein gp62	P23064
	02	Envelope glycoprotein gp62	P0C212
	03	Envelope glycoprotein gp62	Q03816
	04	Envelope glycoprotein gp62	Q03817
	05	Envelope glycoprotein gp62	P14075
	06	Envelope glycoprotein gp62	P03381
HTLV-2	01	Envelope glycoprotein gp62	P03383
HTLV-3	01	Envelope glycoprotein gp62	Q0R5Q9
	02	Envelope glycoprotein gp62	Q09SZ7

### 3.2. Epitope mapping for vaccine construction

The vaccine development process included the prediction of T-cell and B-cell epitopes, as well as the assessment of their biophysical characteristics. Subsequently, the epitopes underwent an evaluation to determine their high antigenicity, non-allergenicity, non-toxicity, conservancy across selected strains, and dissimilarity to the human proteome. Those epitopes meeting these criteria were ultimately selected. Additionally, HTL epitopes were further evaluated for their ability to elicit cytokines, and those that could induce at least one cytokine were included in the vaccine. A list of potential CTL, HTL, and LBL epitopes is provided in **S2 Table in S1 File**. Eventually, 8 CTL, 7 HTL, and 2 LBL epitopes were chosen based on the stringent criteria mentioned in **S3 Table in S1 File** for vaccine construction. Specific linkers and adjuvants were used to conjugate the epitopes, and the vaccine designs were subjected to rigorous testing to confirm their high antigenicity, non-allergenicity, and non-toxicity. **Fig 1A and 1B** illustrate schematic and constructive representations of vaccine construct-1 and 2, respectively, and the conservancy of the epitopes among the selected viral strains is shown in **Fig 2**.

**Fig 1:** Schematic and constructive representation of (A) vaccine construct 1 and (B) vaccine construct 2.

The article "An immunoinformatics and extended molecular dynamics approach for designing a polyvalent vaccine against multiple strains of Human T-lymphotropic virus (HTLV)" was retracted in 2025. Reasons: unreliable results or conclusions; concerns about the peer review; concerns about the article.

**Fig 2:** The multiple sequence alignment analysis demonstrating the conservation of the selected epitopes across various strains and isolates of HTLV. The red boxes highlight the presence of these epitopes in multiple HTLV strains, indicating their conserved nature.

### 3.3. Analyses of the biophysical and structural properties of the vaccine

According to biophysical analyses, vaccine construct-1 and 2 displayed favorable qualities such as solubility, stability, and suitability for further examination (as shown in **S4 Table in S1 File**). Secondary structure analysis of the vaccine designs indicated that random coil was the most prevalent structure. Afterward, 3D structures of the vaccine constructs were generated, which were subsequently refined and validated. The ERRAT value of vaccine construct-1 and vaccine construct-2 were 75 and 95.238 while the Z score were -4.68 and -4.37 respectively. The Ramachandran plot revealed that most residues for both vaccine designs (84.2% for vaccine construct-1 and 89.5% for vaccine construct-2) were in the favored region. The physicochemical property analysis revealed that vaccine construct-2 has better theoretical Isoelectric point (9.55vs9.63), Aliphatic index (71.60vs73.00), GRAVY (-0.156vs -0.233), and other characteristics in comparison to vaccine construct-1. The overall biophysical and structural characteristics of the vaccines indicated that vaccine construct-2 was more appropriate for further analysis. The 3D model and validation of both vaccine constructs can be found in **Fig 3**, while additional information on the secondary structure of the vaccine constructs is provided in **S5 Table and S2 Fig in S1 File**.

**Fig 3:** Structure prediction and validation of vaccine construct 1 (A) 3D model (B) Ramachandran layout and (C) The ERRAT quality value (D) Z score graph, and vaccine construct 2 (E) 3D model (F) Ramachandran layout and (G) The ERRAT quality value (H) Z score graph.

### 3.4. Molecular docking analyses

To assess the interaction between vaccine epitopes and their corresponding MHC-I alleles, we performed the molecular docking analysis. Since vaccine construct-2 exhibited more promising results in terms of biophysical and structural properties, we specifically focused on conducting the analysis using the CTL epitopes chosen to design vaccine construct-2 and their respective MHC-I alleles. **S6 and S7 Tables in S1 File** present the list of epitopes, along with their interacting alleles and docking scores obtained from this analysis. Most of the potential T-cell epitopes exhibited strong binding affinities against both the HLA-A*11:01 and HLA-DRB1*04:01 alleles, as shown in **Fig 4**. Afterward, molecular docking analysis was also conducted to assess the binding affinity of both vaccine constructs with TLR2 and TLR4. The results revealed that vaccine construct-2 had a significantly higher free binding energy and demonstrated a greater docking score with both TLR2 and TLR4. The docking scores obtained from ClusPro and H-dock servers can be found in **Table 2 and S8 Table in S1 File**, respectively. Based on the assigned docking score, solubility, and other desired criteria, vaccine construct-2 was selected for additional Molecular Dynamics (MD) simulations using the Gromacs 2020.4 package to further evaluate its interaction and binding affinity with TLR2 and TLR4 (Berendsen, 1995) [43].

The article "An immunoinformatics and extended molecular dynamics approach for designing a polyvalent vaccine against multiple strains of Human T-lymphotropic virus (HTLV)" was retracted in 2025. Reasons: unreliable results or conclusions; concerns about the peer review; concerns about the article.

**Fig 4:** Docked complexes of HTLV-vaccine epitopes. Docked vaccine epitope sequences A) CPYLGCQSW, B) EVSRLNINL, C) FLNTEPSQL, D) GSMSLASGK, E) IPWKSKLLTL, F) REALQTGITL, and G) VSRLNINLHF. (I: HLA-A, II: HLA-DRB; chains of HLA are shown in different colored ribbons, Chain A: Light brown, Chain B: Light green, chain D: Shade of khakhi, chain E: Light pink, and vaccine epitopes are shown in light blue ribbon and stick representation).

**Table 2:** Binding affinity between Vaccine molecules and TLRs by ClusPro server.

TLR’s	Vaccine	ClusPro docking energy
TLR2	V1	-763.3
	V2	-1018.7
TLR4	V1	-869.6
	V2	-1054.1

### 3.5. Molecular dynamics simulation studies

#### 3.5.1. Root mean square deviation evaluation

The RMSDs in the C-α atom were analyzed independently for each chain of TLRs and vaccine chain. In the TLR2-vaccine complex, chain D has more fluctuations throughout the simulation period with an average of 0.390 nm (**Fig 5A, Table 3**), however, reaching beyond 0.5 nm occasionally. Chain A has a slightly higher RMSD after around 50 ns than chains B and C. The average RMSD for chain A is 0.351 nm, slightly higher than the average RMSD of 0.314 nm for chain C. Chain B has the lowest average RMSD of 0.291 nm with slightly higher deviations during 50–70 ns which is stabilized thereafter. The RMSD for the vaccine chain is slightly higher during the first 10 ns simulation period reaching a maximum of 0.4 nm. Thereafter the RMSD almost remained stable until 90 ns with an average of 0.299 nm and rose to 0.5 nm during the last 10 ns simulation period. In the case of the TLR4-vaccine complex, chains C and D almost stabilize after around 15 ns with an average RMSD of 0.288 and 0.260 nm, respectively (**Fig 5B**). Chain A has initially has low deviations until about 55 ns which rises to around 0.5 nm till 70 ns and again stabilizes with lower RMSD with an overall average RMSD of 0.265 nm. Chain B has deviations after approximately 10 ns with an average of 0.316 nm. The vaccine chain bound to TLR4 has significant deviations until the 60 ns simulation period and stabilized thereafter until the end of the simulation period with an average of 0.344 nm.

The article "An immunoinformatics and extended molecular dynamics approach for designing a polyvalent vaccine against multiple strains of Human T-lymphotropic virus (HTLV)" was retracted in 2025. Reasons: unreliable results or conclusions; concerns about the peer review; concerns about the article.

**Fig 5:** The RMSD analysis. A) RMSD plot for TLR2 chains and bound vaccine chain, and B) RMSD plot for TLR4 chains and bound vaccine chain (color scheme is same as A). The RMSF in side chain atoms of residues. C) RMSF in TLR2 chains and bound vaccine chain, and D) RMSF in TLR4 chains and bound vaccine chain.

**Table 3:** Estimates of averages for different MDS analysis parameters.

	Average (nm)		
	RMSD in C-α atoms	RMSF	Gyrate
TLR2 (Chain A)	0.351 (0.076)	0.176 (0.078)	3.106 (0.045)
TLR2 (Chain B)	0.294 (0.051)	0.149 (0.060)	3.064 (0.024)
TLR2 (Chain C)	0.314 (0.044)	0.137 (0.055)	3.093 (0.022)
TLR2 (Chain D)	0.390 (0.055)	0.157 (0.067)	3.110 (0.031)
Vaccine chain bound to TLR2	0.299 (0.061)	0.219 (0.084)	1.130 (0.023)
TLR4 (Chain A)	0.265 (0.053)	0.169 (0.073)	3.191 (0.049)
TLR4 (Chain B)	0.316 (0.057)	0.154 (0.085)	3.189 (0.027)
TLR4 (Chain C)	0.288 (0.053)	0.160 (0.062)	1.576 (0.010)
TLR4 (Chain D)	0.260 (0.035)	0.127 (0.061)	1.544 (0.010)
Vaccine chain bound to TLR4	0.344 (0.049)	0.258 (0.099)	1.131 (0.034)

Standard deviations in average values are given in parentheses.

#### 3.5.2. Root mean square fluctuation evaluation

Root mean square fluctuations (RMSF) were also analyzed separately for each chain of TLRs and respective bound vaccines. The four chains of TLR2 have almost similar lengths and showed nearly equal magnitude fluctuations (**Fig 5C**). All four chains showed a slightly higher magnitude of fluctuations rising beyond 0.5 nm in the residues 225–250 and 275–325. Further, chain A has comparably higher fluctuations in the first 125 residues. The average RMSF for these four chains is in the range from 0.157 to 0.176 nm. In the case of the bound vaccine, almost all the residues have slightly higher RMSF with an average of 0.219 nm.

Chain A and chain B of TLR4 are equal in length and showed almost similar and lower RMSF with averages of 0.169 and 0.154 nm, respectively (**Fig 5D**). Chain C and D of TLR4 are similar and shorter in length, and slightly more significant fluctuations are seen in chain C residues with an average RMSF of 0.160 nm. The vaccine chain bound to TLR4 similarly has a more considerable fluctuation with an average of 0.258 nm.

#### 3.5.3. Radius of gyration evaluation

The total radius of gyration (Rg) of TLR2 showed that almost all TLR2 chains have a stable Rg in the range of 3.064 to 3.110 nm, where chain B showed a lower Rg amongst all TLR2 chains (**Fig 6A**). Chain A and D have higher Rg with averages of 3.106 and 3.110, respectively. The bound vaccine showed a slightly higher Rg during the first 10 ns simulation period, which stabilizes to a stable Rg with an average of 1.130 nm.

The article "An immunoinformatics and extended molecular dynamics approach for designing a polyvalent vaccine against multiple strains of Human T-lymphotropic virus (HTLV)" was retracted in 2025. Reasons: unreliable results or conclusions; concerns about the peer review; concerns about the article.

**Fig 6:** Radius of gyration analysis. A) Rg in TLR2 chains (left hand panel) and vaccine chain (right hand panel), and B) Rg in TLR4 chain A and B (left hand panel) and TLR4 chain C, chain D vaccine chain (right hand panel).

The chain A and B of TLR4 (part of ectodomain) showed average Rg of 3.191 and 3.189 nm, respectively (**Fig 6B**), where the Rg of chain B almost remained stable throughout the simulation. The attached chains C and D (lymphocyte antigenic units) showed slightly lower Rg, both stable throughout the simulation with average of 1.576 and 1.544 nm, respectively. The bound vaccine chain showed slight fluctuation until the first 50 ns simulation which stabilized to the lowest Rg with an average of 1.131 nm.

#### 3.5.4. Hydrogen bond analysis

The interchain hydrogen bonds between the vaccine and TLR chains were analyzed. The vaccine chain in the case of TLR2 remained bound at the interface of chains C and D, while in the case of TLR4, it remained at the interface of chains B and D. Thus, the hydrogen bonds formed between vaccine chain and chain C and chain D of TLR2 was first investigated (**Fig 7A**). The vaccine chain occupied close contact with TLR2 chain C and an average around 5 hydrogen bonds were found. During the first 25 ns simulation period, an average of around 5 and a maximum of around 10 hydrogen bonds were found, which lowered to average 2 hydrogen bonds till 60 ns and thereafter again around 5 hydrogen bonds re-establish. There is very subtle contact between the vaccine chain and chain D of TLR2 forming only around one hydrogen bond during the first 20 ns simulation period, which rises to around an average of 3 hydrogen bonds until 50 ns. However, after 50 ns until the end of the simulation, an average of around 2 hydrogen bonds were formed.

**Fig 7:** Hydrogen bond analysis plots showing, A) Number of hydrogen bonds formed between TLR2 chain C and vaccine chain (left hand panel) and TLR2 chain D and vaccine chain (right hand panel), and B) Number of hydrogen bonds formed between TLR4 chains B and vaccine chain (left hand panel) and TLR4 chains D and vaccine chain (right hand panel).

Chain B of TLR4 was found in close contact with the vaccine chain and formed around 7 interchain hydrogen bonds during the first 20 ns simulation period reaching a maximum of 10 hydrogen bonds (**Fig 7B**), however, after 20 ns average of only 3 hydrogen bonds formed consistently until the end of the simulation. An average of one interchain hydrogen bond is formed between chain D and the vaccine chain reaching 2 occasionally and reaching a maximum of 5 hydrogen bonds at around 50 ns simulation period.

The article "An immunoinformatics and extended molecular dynamics approach for designing a polyvalent vaccine against multiple strains of Human T-lymphotropic virus (HTLV)" was retracted in 2025. Reasons: unreliable results or conclusions; concerns about the peer review; concerns about the article.

The interchain hydrogen bonds formed were visually inspected to investigate important residues of the vaccine chain involved in hydrogen bond formation. The results of this investigation from the equilibrated trajectory and trajectories captured at 25, 50, 75, and 100 ns are briefly presented here. The equilibrated trajectory of TLR2-vaccine complex showed hydrogen bonds between residues Gly1, Ile2, Ile3, Thr5, Leu6, Lys8, Tyr9, Arg12, Val13, Arg14, Thr35, Arg42, and Lys45 of vaccine chain and chain C residues Asp323, Phe322, Asp235, Thr288, Phe325, and Ser329 and chain D residues Asp327, Glu383, Asp384, Asp235, Glu264, Thr236, Leu354, and Gln357 (**Fig 8A**). Except for the hydrogen bond between Lys45 of the vaccine chain and Glu264 of chain C, most of these hydrogen bonds are transient, and the trajectory at 25 ns showed that the residues Gly1, Ile3, Asn4, Gln7, Lys32, Thr35 of the vaccine form a hydrogen bond with different residues of chain C *viz*. Asn294, Ser298, Phe325, and chain D residues *viz*. Asn294, Ile304, Ser329, Asn297, and Asp299 (**Fig 8B**). The trajectory at 50 ns showed that the hydrogen bond between the residues Gly1, Asn4, Thr35, and Lys45 from vaccine chain and chain C residue Glu264, and chain D residues Asn294, Ile304, and Asp299 remained stable with no new hydrogen bonds (**Fig 8C**). The trajectories captured at 75 ns showed that the residues Thr10, Lys32, and Lys45 from the vaccine chain form a hydrogen bond with chain C residue Asn294, Ser298, and Asp299 and chain D residue Asp299 (**Fig 8D**). The trajectory at 100 ns showed these hydrogen bonds remained intact. However, new hydrogen bonds were formed between vaccine residues Gly1, Lys8, Thr9, Arg14, and Arg42 and chain C residues Asp327, Gly291, Val292, Gly293 and chain D residue Glu336 (**Fig 8E**).

**Fig 8:** The inter-chain hydrogen bonds between vaccine chain (shown in orange color surface/ribbon/sticks) and two chains of TLR2 *viz*. chain C (shown in olive green surface/ribbon/sticks) and chain D (shown in light brown surface/ribbon/sticks).

In the case of the TLR4-vaccine complex, the initial equilibrated trajectory showed many hydrogen bonds between the vaccine chain and TLR4 B and D chains. The residues Arg12, Arg14, Arg17, Cy**S1**8, Ser22, Lys26, Cys33, Ser34, Arg36, Arg38, Arg43, Lys45, and Thr35 formed a hydrogen bond with chain B residues Arg355, Arg382, Glu425, Glu474, Asp502, Asp428, Glu603, Tyr403, Asp379, Glu336, Asp379, Gln523, Asp550, Ser381, Asp405, Gln547 and chain D residue Gln73 (**Fig 9A**). None of these hydrogen bonds are stable, and a new and lone hydrogen bond was formed between the Arg36 residue of the vaccine and Glu287 of chain B (**Fig 9B**). The trajectory at 50 ns showed hydrogen bonds between residues Thr5, Tyr9, and Ser22 of vaccine chain and chain B residues Gln523, Glu474, and chain D residue Ser141 (**Fig 9C**). The trajectory at 75 ns showed the hydrogen bond between Tyr9, Arg17, and Lys45 of the vaccine chain and Glu474, Glu603 of chain B and Ser141 of chain D (**Fig 9D**). The last 100 ns trajectory showed the hydrogen bonds between the residues Thr5, Lys8, Thr9, Arg17, Lys45 and residues Arg606, Gln523, Glu474, and Glu603 of chain B and Ser141 of chain D (**Fig 9E**).

The article "An immunoinformatics and extended molecular dynamics approach for designing a polyvalent vaccine against multiple strains of Human T-lymphotropic virus (HTLV)" was retracted in 2025. Reasons: unreliable results or conclusions; concerns about the peer review; concerns about the article.

**Fig 9:** The inter-chain hydrogen bonds between vaccine chain (shown in orange color surface/ribbon/sticks) and two chains of TLR4 *viz*. chain B (shown in pink surface/ribbon/sticks) and chain D (shown in light brown surface/ribbon/sticks).

#### 3.5.5. Contact map analysis

In the TLR2 vaccine complex, the vaccine is bound at the interface of chains C and D. While in the TLR4 vaccine complex, the vaccine is bound at the interface of chains B and D. The extent of residue-residue contacts between these TLR chains and the vaccine chain was analyzed through contact map analysis (**Fig 10**).

**Fig 10:** Contact maps constructed for the mean smallest distances between network of residues of TLR2 and vaccine. A) TLR2-vaccine complex, and B) TLR4-vaccine complex (The residue-residue contacts between respective TLR chains and vaccine chain are marked in red circles). Gibb’s free energy landscape. C) TLR2-vaccine complex, and D) TLR4-vaccine complex.

The contact maps show that the TLR2 chain C has a slightly greater number of residue-residue contacts with the vaccine chain than those between chain D and the vaccine chain. More residue-residue contacts were found between TLR4 chain B, and the vaccine chain than those between TLR4 chain D and the vaccine chain (**Fig 10A and 10B**).

#### 3.5.6. Principal component analysis and Gibb’s free energy analysis

Principal component analysis (PCA) and corresponding Gibb’s free energy analysis were performed. Comparably, a large energy basin with the lowest energy was found with the TLR4-vaccine complex (**Fig 10**). Among the two energy basins in the TLR2-vaccine complex, the one occupying the energy range of around -50 kJ mol^-1^ on PC1 and 5 to -15 kJ mol^-1^ on PC2 is the lowest energy basin, while the other one with the higher energy range is beyond 200 kJ mol^-1^ on PC1 and spread across 60 to -30 kJ mol^-1^ on PC2 (**Fig 10C**). The TLR4-vaccine complex has a unique energy basin spread across 10 to -20 kJ mol^-1^ on PC1 and 10 to -10 kJ mol^-1^ on PC2, suggesting a large stable lowest energy conformation (**Fig 10D**).

The article "An immunoinformatics and extended molecular dynamics approach for designing a polyvalent vaccine against multiple strains of Human T-lymphotropic virus (HTLV)" was retracted in 2025. Reasons: unreliable results or conclusions; concerns about the peer review; concerns about the article.

#### 3.5.7. Dynamic cross-correlation (DCC) analysis

Through DCC analysis, the time-correlated information of inter-chain and intra-chain residue to residue contacts and motions was analyzed. In DCC plots, the color gradient ranges from blue (negative correlation, less likely) to red (positive correlation, more evident) corresponding to the correlation coefficients -1 and +1, respectively, and the lighter shades indicate weaker correlations, where the white color indicates no correlation. The DCC correlation of the vaccine chain with each chain of TLRs was analyzed (**Fig 11A and 11B**). The results for the TLR2-vaccine complex indicate that the residues from chains B, C, and D are positively correlated with the vaccine chain with a stronger correlation with chains B and C. Similarly, in the TLR4-vaccine complex, chains B, C, and D have moderate to strong positive correlation with vaccine chain.

**Fig 11:** DCC analysis for vaccine chain complex with A) TLR2, and B) TLR4. (The plot of DCCM shows residue-wise correlation in each complex. The separation of TLR chain and vaccine chain is shown at the bottom of each plot). DSSP plots for individual TLR chains and corresponding vaccine chain. C) TLR2-vaccine complex and D) TLR4-vaccine complex.

#### 3.5.8. DSSP analysis

The secondary structural changes during MD simulation were analyzed from DSSP analysis. Mainly, the TLR chains which are in close contact with vaccine chains were analyzed. The results showed that the TLR2 chains C and D are relatively stable for secondary structural changes (**Fig 11C and 11D**). However, the vaccine chain showed significant structural changes in the loop regions. Similarly, chains B and D of TLR4 showed relatively stable secondary structure, while the vaccine chain bound to TLR4 showed numerous secondary structural changes in the loop regions.

#### 3.5.9. MM-PBSA calculation

The MM-PBSA calculations on 10 trajectories isolated, each isolated at 10 ns, for every complex. MM-PBSA calculations estimated the interaction energies viz. van der Waal energy, electrostatic energy, polar solvation energy, SASA energy, and binding energy (ΔGbinding) between TLR chains and vaccine chain (**Table 4**). The results show that the TLR4-vaccine complex has more favorable binding energy than the TLR2-vaccine complex. The lower electrostatic, van der Waal, and polar solvation energy for the TLR4-vaccine complex might be responsible for the lower and favorable binding free energy.

**Table 4:** Results of MM-PBSA calculations.

Complex with vaccine	van der Waal energy (kJ mol^-1^)	Electrostatic energy (kJ mol^-1^)	Polar solvation energy (kJ mol^-1^)	Solvent accessible surface area energy (kJ mol^-1^)	Binding energy (ΔG_binding_) (kJ mol^-1^)
TLR2	-345.705 (10.329)	-2174.379 (38.706)	1049.555 (85.192)	-49.017 (1.324)	-1515.803 (51.212)
TLR4	-300.948 (23.796)	-2389.808 (38.261)	879.529 (112.236)	-41.870 (2.628)	-1848.399 (71.663)

Standard deviations are given in parentheses.

The article "An immunoinformatics and extended molecular dynamics approach for designing a polyvalent vaccine against multiple strains of Human T-lymphotropic virus (HTLV)" was retracted in 2025. Reasons: unreliable results or conclusions; concerns about the peer review; concerns about the article.

### 3.6. Disulfide engineering and *in silico* cloning studies

By using the DbD2 server, a total of 7 pairs of amino acid residues for vaccine construct-2 have been discovered as having the ability to structure disulfide bonds. Three pairs of amino acid residues (Cys 11 –Gly 15, Cys 11 –Cys 40, and Cys 18 –Cys 33) were carefully chosen due to their compatibility with standard disulfide bond formation conditions, with energy levels lower than 2.5 Kcal/mol (**S3 Fig in S1 File**). In the codon adaptation study of the vaccine, the codon adaptation index (CAI) revealed that the adapted codons displayed a higher proportion of the most abundant codons. Notably, the optimized codons exhibited a significant GC content of 54.6428 and a CAI of 0.9690. To ensure the safety of the cloning process, the absence of restriction sites for BsgI and AvaI was confirmed. Subsequently, the optimized codons, along with the BsgI and AvaI restriction sites, were inserted into the pET28a (+) vector. This resulted in the generation of a 3515 base pair clone, which included the desired 387 bp sequence, with the remaining portion belonging to the vector. The desired area between the pET28a (+) vector sequence was indicated in red, as depicted in **S4 Fig in S1 File**.

## 4. Discussion

The substantial impact of HTLV viruses in causing a spectrum of inflammatory, immunosuppressive disorders, and cancer underscores the need for urgent preventive and treatment strategies to mitigate their severe consequences. To address this exigency, our study adopted a reverse vaccinology approach [67–69] to create a multi-epitope-based vaccine that specifically targets multiple virulent HTLV subtypes. Moreover, we meticulously analyzed the interactions between the vaccine and Toll-like receptors (TLRs), yielding insights that can steer future research toward effective strategies and countermeasures for HTLV-related diseases or future outbreaks.

Our vaccine design centered on the envelope glycoprotein gp62, a key outer membrane protein containing numerous epitope binding sites crucial for the infectious process and immune response of HTLV [70,71]. Epitope mapping was executed to identify T cell and B cell epitopes, both essential for provoking the host’s immune response to viral infection [72,73]. Utilizing IEDB algorithms, we predicted epitopes with low binding energies, ensuring robust target affinity. The selected epitopes displayed high antigenicity with no allergenicity and toxicity, indicating their potential to evoke a robust and safe immune reaction against the viral infection. Combining the selected T cell and B cell epitopes with suitable linkers, we integrated PADRE and hBD adjuvants to enhance immunogenicity within the human body. The hBD adjuvant attracts immature dendritic cells, naive memory T cells, and monocytes to the infection site, thereby bolstering innate and adaptive host defense mechanisms. Incorporating adjuvants and linkers not only enhances the vaccine’s antigenicity and immunogenicity but also stabilizes the construct, improving its profile and longevity [74].

The article "An immunoinformatics and extended molecular dynamics approach for designing a polyvalent vaccine against multiple strains of Human T-lymphotropic virus (HTLV)" was retracted in 2025. Reasons: unreliable results or conclusions; concerns about the peer review; concerns about the article.

Two vaccines were initially designed with selected epitopes which were highly antigenic, non-allergenic, and non-toxic, confirming safety and immune response effectiveness. However, solubility analysis revealed that Vaccine construct-2 was soluble, while construct 1 was insoluble–an important factor for vaccine efficacy [75]. Both constructs were stable (instability index < 40) and possessed favorable aliphatic index values, indicating stability at human body temperature. Their negative GRAVY value implied higher solubility. Disulfide engineering in construct 2 introduced amino acid pairs for enhanced stability and efficacy [76]. Both vaccine constructs had prominent random coil secondary structures. However, vaccine construct-2 showed a superior structural profile with a higher ERRAT score (95.238 vs. 75) and more structure in the favored region (89.5% vs. 84.2%). Moreover, both constructs had high-quality models with no structure in the disallowed region of the Ramachandran plot. Overall, the structure prediction confirmed that both vaccine constructs have suitable structures and should be adequately stable.

Having established the superiority of vaccine construct-2 in previous comparative analyses, our exclusive focus turned to molecular docking analysis with this particular construct. Our investigation revolved around the molecular interactions between the epitopes of vaccine construct-2 and their corresponding HLA alleles, as well as the interactions between the vaccine and its corresponding TLRs. The initial step involved docking the CTL epitopes of vaccine construct-2 with HLA-A*11:01 and HLA-DRB1*04:01 to assess their binding affinity with representative HLA alleles. Notably, HLA-A*11:01 is a significant human leukocyte antigen, while HLA-DRB1*04:01 is prevalent in patients with severe extra-articular rheumatoid arthritis associated with HTLV [77,78]. These alleles play a pivotal role in presenting viral antigens to T cells, thereby triggering an effective immune response [79]. Evidently, the CTL epitopes exhibited robust binding affinity with both HLA alleles. Subsequent molecular docking was carried out to evaluate the interaction between the vaccine construct and TLR2, as well as TLR4. This analysis was conducted using the ClusPro server and H-dock server. TLR2 and TLR4 are suitable targets for vaccine constructs due to their expression on the cell surface and intracellularly in dendritic cells (DCs), endothelial cells, and epithelial cells (ECs) [80]. Impressively, vaccine construct-2 demonstrated the most favorable docking scores with both TLR2 and TLR4, yielding -1018.7 and -1054.1 respectively in the ClusPro server, and -281.88 and -279.46 respectively in the H-dock server. Guided by the collective results of prior experiments encompassing antigenicity, solubility, physicochemical properties, and binding affinity, the selection of vaccine construct-2 for further molecular dynamic simulation studies was evident.

The article "An immunoinformatics and extended molecular dynamics approach for designing a polyvalent vaccine against multiple strains of Human T-lymphotropic virus (HTLV)" was retracted in 2025. Reasons: unreliable results or conclusions; concerns about the peer review; concerns about the article.

TLR2 has four equally sized chains, namely chain A, B, C, and D. In contrast, TLR4 consists of two chains in the TLR ectodomain, chain A, and chain B, along with two antigen units, chain C and chain D. The highest magnitude of RMSD was observed in chain D of TLR2, while the other three chains showed relatively stable RMSD. Conversely, RMSD in corresponding chains A and B of TLR4 displayed slight deviations throughout the simulation. RMSD in the antigen units of TLR4 (chain C and chain D) remained relatively stable. Furthermore, the RMSD in the vaccine chain bound to TLR2 was lower than that bound to TLR4, indicating the TLR2-vaccine complex’s greater stability.

RMSF analyses demonstrated almost analogous and relatively lower fluctuations in all TLR2 chains, except for residues in the range 200–325, indicating uniform conformational changes in these chains. In contrast, TLR4 ectodomain chains (chains A and B) exhibited analogous and minimal fluctuations in nearly all residues, suggesting a stable conformation. The antigen units (chain C and chain D) in TLR4 showed some fluctuations, with chain D in close contact with the vaccine chain. Both complexes exhibited marginal fluctuations in the non-terminal residues of the vaccine chain, suggesting comparable stability.

All four chains of TLR2 displayed almost similar total Rg, indicating comparable compactness. TLR4 chains A and B also showed similar compactness, indicating analogous and rigid structural features. As short proteins, the antigen units (chain C and chain D) in TLR4 displayed a very compact nature with significantly lower total Rg than TLR4 chains A and B. After approximately 25 ns, the vaccine chains bound to TLR2 and TLR4 showed a very compact nature with stable and lowest total Rg.

The article "An immunoinformatics and extended molecular dynamics approach for designing a polyvalent vaccine against multiple strains of Human T-lymphotropic virus (HTLV)" was retracted in 2025. Reasons: unreliable results or conclusions; concerns about the peer review; concerns about the article.

Hydrogen bond analysis revealed that the vaccine chain in both complexes formed maximum and more consistent hydrogen bonds with chain C in TLR2 and chain B in TLR4. However, the hydrogen bonds between chain D and the vaccine in TLR2 and TLR4 complexes significantly differed, with more hydrogen bonds observed in TLR2. These results suggested that the vaccine chain interacted and formed many key hydrogen bonds with chains C and D of TLR2, compared to the vaccine forming hydrogen bonds with chains B and D of TLR4. The number of non-bonded interactions, such as hydrogen bonds, indicated a better affinity of the vaccine and overall stability of the respective complexes. Based on these grounds, the TLR2-vaccine complex exhibited better stability, with the vaccine construct showing a more favorable affinity for TLR2.

Contact analysis further supported the hydrogen bond analysis, with the TLR2-vaccine complex displaying a more significant number of residue-residue contacts between chain C and chain D of TLR2 and the vaccine chain. In contrast, fewer TLR4 chain B and D residues showed such contact with vaccine residues.

Gibb’s free energy landscapes analysis indicated fewer low-energy conformations in the TLR2-vaccine complex compared to the TLR4-vaccine complex. The latter exhibited a major low energy basin with many lowest energy conformations, indicating a more stable state.

The DCC analysis revealed positively correlated residues from chain B, chain C, and chain D of TLR2 and moderately positive correlations from all chains of TLR4. TLR4-vaccine chain exhibited very few negatively correlated residues, confirming its better stability.

DSSP analysis indicated that chain A and chain D of TLR2, as well as chain B of TLR4, remained stable for any secondary structural changes. However, chain D, the antigen unit in TLR4, showed a few significant secondary structural changes, suggesting its structural flexibility. In both complexes, the vaccine chains underwent secondary structural changes, mainly in the loops or turns, possibly contributing to the vaccine construct’s better and more compact structure.

MM-PBSA analysis suggested that the vaccine construct bound to TLR4 had a more favorable binding affinity than the TLR2-bound vaccine construct. The significant difference in energetics was in the electrostatic energy, with TLR4 showing significantly lower electrostatic energy than TLR2.

In conclusion, molecular dynamics simulations revealed enhanced stability and a favorable affinity in the TLR2-vaccine complex, as supported by contact analysis and secondary structure stability. On the other hand, MM-PBSA analysis favored the TLR4-vaccine complex due to lower electrostatic energy.

The article "An immunoinformatics and extended molecular dynamics approach for designing a polyvalent vaccine against multiple strains of Human T-lymphotropic virus (HTLV)" was retracted in 2025. Reasons: unreliable results or conclusions; concerns about the peer review; concerns about the article.

## 5. Conclusion

The research on the multi-epitope-based vaccine targeting highly virulent subtypes of HTLV has significant future implications. The findings contribute to the development of an effective preventive and therapeutic approach for HTLV-associated disorders. By utilizing a reverse vaccinology strategy, the study demonstrates the design and characterization of vaccine constructs with high antigenicity, safety, and stability. The incorporation of adjuvants and linkers enhances the immunogenicity of the vaccine. Molecular docking studies and molecular dynamic simulations provide insights into the strong binding affinity and stability of the vaccine with key immune receptors, such as HLA alleles, TLR2, and TLR4. These findings lay the foundation for potential strategies to prevent and manage HTLV-related diseases and outbreaks, offering promising prospects for improved clinical outcomes in the future.

## Supporting information

S1 File (PDF)
